The article "Combined application of zinc and iron-lysine and its effects on morpho-physiological traits, antioxidant capacity and chromium uptake in rapeseed (Brassica napus L.)" was retracted in 2022. Reasons: compromised peer review; a conflict of interest; concerns about the authorship.

# Combined application of zinc and iron-lysine and its effects on morpho-physiological traits, antioxidant capacity and chromium uptake in rapeseed (*Brassica napus* L.)

**DOI:** 10.1371/journal.pone.0262140

**Published:** 2022-01-07

**Authors:** Ihsan Elahi Zaheer, Shafaqat Ali, Muhammad Hamzah Saleem, Hafiza Sana Yousaf, Afifa Malik, Zohaib Abbas, Muhammad Rizwan, Muyassar H. Abualreesh, Aishah Alatawi, Xiukang Wang

**Affiliations:** 1 Department of Environmental Sciences and Engineering, Government College University, Faisalabad, Pakistan; 2 Department of Biological Sciences and Technology, China Medical University, Taichung, Taiwan; 3 College of Plant Science and Technology, Huazhong Agricultural University, Wuhan, China; 4 Department of Environmental Sciences, Lahore College for Women University, Lahore, Pakistan; 5 Sustainable Development Study of Center, Government College University, Lahore, Pakistan; 6 Department of Marine Biology, Faculty of Marine Sciences, King Abdualaziz University, Jeddah, Saudi Arabia; 7 Biology Department, Faculty of Science, Tabuk University, Tabuk, Saudi Arabia; 8 College of Life Sciences, Yan’an University, Yan’an, China; Ghazi University, PAKISTAN

## Abstract

Environmental contamination of chromium (Cr) has gained substantial consideration worldwide because of its high levels in the water and soil. A pot experiment using oil seed crop (rapeseed (*Brassica napus* L.)) grown under different levels of tannery wastewater (0, 33, 66 and 100%) in the soil using the foliar application of zinc (Zn) and iron (Fe)–lysine (lys) has been conducted. Results revealed that a considerable decline in the plant growth and biomass elevates with the addition of concentrations of tannery wastewater. Maximum decline in plant height, number of leaves, root length, fresh and dry biomass of root and leaves were recorded at the maximum level of tannery wastewater application (100%) compared to the plants grown without the addition of tannery wastewater (0%) in the soil. Similarly, contents of carotenoid and chlorophyll, gas exchange parameters and activities of various antioxidants (superoxidase dismutase (SOD), peroxidase (POD), catalase (CAT) and ascorbate peroxidase (APX)) were also reduced significantly (*P* < 0.05) with the increasing concentration of tannery wastewater (33, 66 and 100%) in the soil. In addition, a combined application of Zn and Fe-lys reduced the accumulation and uptake of toxic Cr, while boosting the uptake of essential micronutrients such as Zn and Fe in different tissues of the plants. Results concluded that exogenous application of micronutrients chelated with amino acid successfully mitigate Cr stress in *B*. *napus*. Under field conditions, supplementation with these micronutrient-chelated amino acids may be an effective method for alleviating metal stress in other essential seed crops.

The article "Combined application of zinc and iron-lysine and its effects on morpho-physiological traits, antioxidant capacity and chromium uptake in rapeseed (Brassica napus L.)" was retracted in 2022. Reasons: compromised peer review; a conflict of interest; concerns about the authorship.

## 1. Introduction

Contamination of soil with potentially toxic elements (PTEs) is a pressing and complex problem intensely felt worldwide, particularly in densely industrialized and populated areas [1–4]. Rapid growth of industries and manufacturing operations like smelting, melting, electroplating and mechanical set-ups leads to the extensive contamination of soil with contaminates like abovementioned PTEs [5–8]. However, anthropogenically origin sources related to the metal-enriched sewage sludges in agriculture, combustion, livestock manures, application of metal-based pesticides, electronics (manufacture, use, and disposal), volcanic eruptions, forest fires, industrial processes, municipal wastes, and agricultural activities [9, 10]. Extreme accumulation of PTEs in arable soil not only causes pollution of aquatic and terrestrial environments, but also escalates the likelihoods of human exposure with PTEs [3]. Copious public health distress rises if food products grown on such polluted soil come into national markets, which ultimately exposes of the wider population to PTEs contamination [11].

In Pakistan, aquifers have already been exhausted due to injudicious consumption of groundwater for irrigation purpose to produce crops and fodder [12–14]. So, there is a need to investigate some approaches to reduce the necessity of potable water in this sector. Reuse of wastewater as a renewable resource for irrigation can be a sustainable approach to mitigate the ever-increasing irrigation caused water scarcity around the globe [15, 16]. Nevertheless, depending upon the wastewater resources, it may contain non-biodegradable pollutants such as lead, cadmium, chromium, nickel, copper, zinc, mercury, and arsenic [17].

Prompt industrial and economic developments throughout the world has led to a range of environmental concerns including the contamination of soil with toxic PTEs [18, 19]. Rapid industrialization is causing water pollution as most of the wastewater is being dumped unprocessed back into the water system [20, 21]. Farmers are using wastewater for irrigation, especially in suburban areas to overcome the shortage of canal water [22–24]. Furthermore, wastewater also contains many nutrients which results in an increase in plant growth and productivity and may also reduce the need of excessive use of artificial fertilizers [25–27]. Besides having the several benefits of wastewater for agricultural crop production, it may contain many organic and inorganic contaminants which may deteriorate the quality of crops depending upon plant species and type of contaminant [19, 28]. Among different types of wastewater, tannery wastewater is being produced owing to the increase in the tanning industry in Pakistan and worldwide [3]. Tannery wastewater is used for the growth of crops, especially vegetables which may contaminate food with toxic metals, mainly chromium (Cr) [25, 26].

The article "Combined application of zinc and iron-lysine and its effects on morpho-physiological traits, antioxidant capacity and chromium uptake in rapeseed (Brassica napus L.)" was retracted in 2022. Reasons: compromised peer review; a conflict of interest; concerns about the authorship.

Cr is a potentially noxious metal and it does not have any vital function in metabolic activities of plants [29]. Industrial process (tanning effluents) along with natural and anthropogenic activities result in amplified accumulation of chromium in surrounding environments [18, 30]. Excess Cr in plants may cause toxic effects in plants and reduces growth, photosynthesis, mineral nutrients adsorption, and quality [31]. Combustion of oil, coal and waste from chemical, metallurgy and tannery industrial effluents adds 2,000–5,000 mg Cr L^–1^ in contrast to the acceptable limit of 2 mg Cr L^–1^, which degrade the soil through excessive uptake of Cr [32]. Higher Cr levels in plants cause ultra–structural alteration, oxidative stress in plants and increased electrolyte leakage (EL), malondialdehyde (MDA) concentrations, and induces alterations in antioxidant enzyme activities such as superoxide dismutase (SOD), peroxidase (POD) and catalase (CAT) and ascorbate peroxidase (APX) [33–36]. Hence, it is required to safeguard plants from Cr toxicity to counter the phytotoxicity and oxidative stress triggered by the uptake of Cr in plants.

In the world, rapeseed (*Brassica napus* L.) is considered as essential oilseed crop and is regarded as the second major source of vegetable oil after soybean [37, 38]. Oil rapeseed (*B*. *napus*) has a tremendous capacity to combat the stress induced by the PTEs’ toxicity [39, 40]. Among different PTEs, contamination of Cr has shown noticeable influence on growth, ultra-structural, physicochemical and molecular profiling of the *B*. *napus* [41]. *B*. *napus* can tolerate various kinds of PTEs stresses, owing to its physiological and biological processes, and it also has the capacity to withstand chromium stress [15, 41].

To date, many scientific approaches have been employed to remediate the PTEs stress in plants, particularly by using exogenous applied amino acids. Amino acids play a very critical role in metal compartmentation, transport and tolerance in plants. Zinc (Zn) and iron (Fe) chelated fertilizers complexed with lysine (lys) as amino acid have been reported to improve the growth and yield of crops [42, 43]. Fruitful application of micronutrients expressively mitigates the toxic effects of PTEs stress in plants [44, 45]. Both Fe and Zn are important micronutrients as they play a very critical role in various metabolic processes in plants including photosynthesis, DNA synthesis and respiration [23]. Zn chelated with the amino acid lys effectively mitigates the Cr stress in *Oryza sativa* and *S*. *oleracea* and improved the growth of plant through Zn fortification [22, 46]. Similarly, a previous study reported that Fe-lys can be effectively used as operative amendment in the reduction of Cd stress in *Oryza sativa* [47]. However very little is known about the role of both Zn and Fe-lys regarding the mitigation of PTEs stress in pants.

The article "Combined application of zinc and iron-lysine and its effects on morpho-physiological traits, antioxidant capacity and chromium uptake in rapeseed (Brassica napus L.)" was retracted in 2022. Reasons: compromised peer review; a conflict of interest; concerns about the authorship.

There are various studies about the application of Zn and Fe-lys on different crops under range of PTEs stresses [11, 22, 46, 47], where there is no significant literature present on the combined application of Zn and Fe-lys on crops. This study aims to address this issue and to add knowledge about (i) the role of Zn and Fe–lys on plant growth, fresh weights, dry weights, chlorophyll contents, gas exchange characteristics, oxidative stress and antioxidant response and (ii) uptake and accumulation of Fe, Zn and Cr in different parts of *B*. *napus* when cultivated with wastewater rich in Cr concentration. To the best of our knowledge, this study is among the few studies which focuses on the metal tolerance and accumulation among oil seed crops in order to investigate their suitability for metal–contaminated sites. Findings from the present study will add to our understanding of the mechanism of Cr tolerance and accumulation in *B*. *napus* with the foliar application of Zn and Fe–lys.

## 2. Material and methods

### 2.1 Description of site and soil sampling

Soil surface samples (0-22cm) were carefully taken from the botanical garden, Department of Botany, University of Punjab Lahore, Pakistan (31.4015° N, 74.3070° E). Soil samples were crushed softly with hands, and all visible portions of dead and flourishing vegetation along with other dirt particles were detached at the site. The soil samples were air dried. Debris and mud particles were removed from the dried soil using a 2-mm sieve. All samples of soil were kept in plastic bags at were stored at room temperature.

### 2.2 Determination of soil and wastewater physico-chemical characteristics

Total organic content of the soil was estimated via subsequent titration and dichromate oxidation with ferrous ammonium sulfate according to the method describe by Walkley and Black [48]. Similarly, ion concentration in the soil, sodium adsorption ratio (SAR) and electrical conductivity (EC) were also carefully estimated with the method given by Page [49]. Soil sampling was performed with the assistance of ammonium bicarbonate diethylenetriamine penta acetic acid (AB-DTPA) solution for the appropriate measurement of extractable trace elements [50]. Physiochemical characteristics of the soil under study are given in S1 Table. Tannery wastewater used in this study was carefully collected from tannery industries located in Kasur, Punjab Pakistan. Physiochemical features of tannery wastewater used in the study were carefully estimated according to the set APHA protocols given for the estimation of water and wastewater. Comprehensive details of major characteristics of tannery wastewater used in this experiment are presented in S2 Table.

The article "Combined application of zinc and iron-lysine and its effects on morpho-physiological traits, antioxidant capacity and chromium uptake in rapeseed (Brassica napus L.)" was retracted in 2022. Reasons: compromised peer review; a conflict of interest; concerns about the authorship.

### 2.3 Experimental design

The present experimental work was conducted in the wire house Department of Botany, the University of the Punjab Lahore, Pakistan (31.4015° N, 74.3070° E), from an average depth of 0–15 cm, in an open environment, protected from human and animal interactions. The plants were protected from rainfall by covering the whole wire house with a plastic sheet. The pots used in this study were rotated regularly in order to avoid environmental effects on the plants and to avoid any effect of phototropism on the plants due to sunlight. Seeds of rapeseed (*Brassica napus* L.) (cv. Faisal canola) were collected from Ayub Agricultural Research Institute Faisalabad, Pakistan (31.4041°N, 73.0487°E). The seeds were surface sanitized with H_2_O_2_ solution and washed 5 times with distilled water before sowing in pots. *B*. *napus* seeds were uniformly sowed in plastic pots which was filled with 5 kg of soil. Experiments were conducted accordingly with completely randomized design (CRD) and with three replicates of each treatment. After a germination time of two weeks, *B*. *napus* seedling were treated with the foliar application of Zn and Fe-lys (Zn–lys 0, 10 mg/L and Fe–lys 0, 5 mg/L) along with treatment of tannery wastewater with different levels (0, 33, 66 and 100%). Irrigation with tannery wastewater was supplied once in a week. In addition, application of Zn and Fe-lys was also supplied once a week with a volume of one liter for each spray. We have used 4 L of Zn and Fe-lys in the whole experiment which was sprayed at 4 different intervals of the experiment. However, the controls grown without the application of Zn and Fe-lys was sprayed with the distilled water. In order to mitigate the crucial deficiency of macronutrients, potassium sulphate (SOP) and phosphate were carefully applied to plants as fertilizer by following the methodology described by Bashir et al. [47].

### 2.4 Treatments

Eight treatments regarding wastewater and Fe and Zn-lys applications was used for this study. A detailed description of these treatments are as follow; T1(control): tannery wastewater 0%, Zn-lys 0 and Fe-lys 0 mg/ L, T2: tannery wastewater 0%, Zn-lys 10 and Fe-lys 5 mg/ L, T3: tannery wastewater 33%, Zn-lys 0 and Fe-lys 0 mg/ L, T4: tannery wastewater 33%, Zn-lys 10 and Fe-lys 5 mg/ L, T5: tannery wastewater 66%, Zn-lys 0 and Fe-lys 0 mg/ L, T6: tannery wastewater 66%, Zn-lys 10 and Fe-lys 5 mg/ L, T7: tannery wastewater 100%, Zn-lys 0 and Fe-lys 0 mg/ L, T8: tannery wastewater 100%, Zn-lys 10 and Fe-lys 5mg/L.

The article "Combined application of zinc and iron-lysine and its effects on morpho-physiological traits, antioxidant capacity and chromium uptake in rapeseed (Brassica napus L.)" was retracted in 2022. Reasons: compromised peer review; a conflict of interest; concerns about the authorship.

### 2.5 Plant harvesting

60 days after sowing (DAS), plants were harvested and rinsed thoroughly with normal tap water to wash off the aerial deposition and then cautiously separated into roots and shoots. All plants were rooted up allowing to study different morpho-physiological traits in late December 2017. The sampled leaves were washed with distilled water, immediately placed in liquid nitrogen, and stored in a freezer at low temperature (−80°C) for further analysis. Three plants per treatment were selected randomly for morphological studies. Several leaves were counted, and the plant height (cm) was recorded from the root neck to the upper most part of the shoot. The leaf area was measured by using a leaf area meter (LI-2000, LI-COR, USA). Leaves and roots fresh biomass was measured by weighing. Later, leaves and roots were dried in an oven at 105°C for 1 h, then at 70°C for 72 h allowing to determine the dry weight. Roots were immersed in 20 mM Na_2_EDTA for 15–20 min to remove Cr adhered to the surface of the roots. Then, roots were washed thrice with distilled water and finally once with de-ionized water and dried for further analysis.

### 2.6 Determination of chlorophyll contents and gas exchange parameters

For chlorophyll content analysis, 0.1 g of fresh leaf sample was extracted with 8 mL of 95% acetone for 24 h at 4°C in the dark. The absorbance was measured by a spectrophotometer (UV-2550; Shimadzu, Kyoto, Japan) at 646.6, 663.6 and 450 nm. Chlorophyll content was calculated by the standard method of Arnon [51].

Net photosynthesis (P*n*), leaf stomatal conductance (g*s*), transpiration rate (T*s*), and water use efficiency (WUE) were measured from three different plants in each treatment group. On the same day (before sampling) these parameters were measured in between 11:30 and 13:30 with a clear sky. Rates of leaf P*n*, g*s*, T*s*, and C*i* were measured with an LI–COR gas–exchange system (LI-6400; LICOR Biosciences, Lincoln, NE, USA) with a red-blue LED light source on the leaf chamber. In the LI-COR cuvette, CO_2_ concentration was set as 380 mmol mol^–1^ and LED light intensity was set at 1000 mmol m^–2^ s –^1^, which is the average saturation intensity for photosynthesis in *B*. *napus* [52].

The article "Combined application of zinc and iron-lysine and its effects on morpho-physiological traits, antioxidant capacity and chromium uptake in rapeseed (Brassica napus L.)" was retracted in 2022. Reasons: compromised peer review; a conflict of interest; concerns about the authorship.

### 2.7 Determination of oxidative stress indicators

The degree of lipid peroxidation was evaluated as malondialdehyde (MDA) content. Briefly, 0.1 g of frozen leaves were ground at 4°C in a mortar with 25 mL of 50 mM phosphate buffer solution (pH 7.8) containing 1% polyethene pyrrole. The homogenate was centrifuged at 10,000 × g at 4°C for 15 min. The mixtures were heated at 100°C for 15–30 min and then quickly cooled in an ice bath. The absorbance of the supernatant was recorded by using a spectrophotometer (xMark™ microplate absorbance spectrophotometer; Bio-Rad, United States) at wavelengths of 532, 600 and 450 nm. Lipid peroxidation was expressed as l mol g^−1^ using the following formula: 6.45 (A532−A600) − 0.56 A450. Lipid peroxidation was measured using a method previously published by Health and Packer [53].

To estimate H_2_O_2_ content of plant tissues (leaf samples), 3 ml of sample extract was mixed with 1 ml of 0.1% titanium sulphate in 20% (v/v) H_2_SO_4_ and centrifuged at 6,000 g for 15 min. The yellow colour intensity was evaluated at 410 nm. The H_2_O_2_ level was computed by extinction coefficient of 0.28 mmol^−1^ cm^−1^. The contents of H_2_O_2_ were measured by following the method of Jana and Choudhuri [54].

Stress-induced electrolyte leakage (EL) of uppermost stretched leaves was determined by Dionisio-Sese and Tobita [55] method. The leaves were cut into minor slices (5 mm length) and placed in test tubes having 8 mL distilled water. These tubes were incubated and transferred into water bath at 32°C for 2 h prior to measuring the initial electrical conductivity (EC_1_). The samples were autoclaved at 121°C for 20 min, and then cooled down to 25°C before measuring the final electrical conductivity (EC_2_). Electrolyte leakage was measured using pH/conductivity meter (model 720, INCO-LAB Company, Kuwait) and calculated as:

EL = (EC_1_/ EC_2_) = × 100

### 2.8 Determination of activities of antioxidant enzymes

To evaluate enzyme activities, fresh leaves (0.5 g) were homogenized in liquid nitrogen and 5 mL of 50 mmol sodium phosphate buffer (pH 7.0) including 0.5 mmol EDTA and 0.15 mol NaCl. The homogenate was centrifuged at 12,000 × g for 10 min at 4°C, and the supernatant was used for the measurements of superoxidase dismutase (SOD) and peroxidase (POD) activities. SOD activity was assayed in 3 mL reaction mixture containing 50 mM sodium phosphate buffer (pH 7), 56 mM nitro blue tetrazolium, 1.17 mM riboflavin, 10 mM methionine and 100 μL enzyme extract. Finally, the sample was measured by using a spectrophotometer (xMark™ microplate absorbance spectrophotometer; Bio-Rad). Enzyme activity was measured using a method by Chen and Pan [56] and expressed as U g^−1^ FW.

The article "Combined application of zinc and iron-lysine and its effects on morpho-physiological traits, antioxidant capacity and chromium uptake in rapeseed (Brassica napus L.)" was retracted in 2022. Reasons: compromised peer review; a conflict of interest; concerns about the authorship.

Peroxidase (POD) activity in the leaves was estimated using the method of Sakharov and Ardila [57], using guaiacol as the substrate. A reaction mixture (3 mL) containing 0.05 mL of enzyme extract, 2.75 mL of 50 mM phosphate buffer (pH 7.0), 0.1 mL of 1% H_2_O_2_ and 0.1 mL of 4% guaiacol solution was prepared. Increases in the absorbance at 470 nm because of guaiacol oxidation was recorded for 2 min.

Catalase (CAT) activity was analyzed according to Aebi [58]. The assay mixture (3.0 mL) was comprised of 100 μL enzyme extract, 100 μL H_2_O_2_ (300 mM) and 2.8 mL 50 mM phosphate buffer with 2 mM ETDA (pH 7.0). The CAT activity was measured from the decline in absorbance at 240 nm as a result of H_2_O_2_ loss (ε = 39.4 mM^−1^ cm^−1^).

Ascorbate peroxidase (APX) activity was measured according to Nakano and Asada [59]. The mixture containing 100 μL enzyme extract, 100 μL ascorbate (7.5 mM), 100 μL H_2_O_2_ (300 mM) and 2.7 mL 25 mM potassium phosphate buffer with 2 mM EDTA (pH 7.0) was used for measuring APX activity. The oxidation pattern of ascorbate was estimated from the variations in wavelength at 290 nm (ε = 2.8 mM^−1^ cm^−1^).

### 2.9 Determination of Fe, Zn and Cr concentrations in plant

Digestion of plant samples was carried out through di−acid (HNO_3_−HClO_4_) method. Dry samples (0.5 g) of both roots and leaves were added in a flask having 10 mL of HNO_3_−HClO_4_ (3:1, v:v), and the mixture was kept overnight. After that, 5 mL HNO_3_ was added and samples were completely digested by placing on a hot plate [60]. Contents of Fe, Zn and Cr in roots and shoots of the plants was measured by using an atomic absorption spectrophotometer.

### 2.10 Statistical analysis

The normality of data was analyzed using IBM SPSS software (Version 21.0. Armonk, NY, USA: IBM Corp) through a multivariate post hoc test, followed by a Duncan’s test in order to determine the interaction among significant values. Testing showed that all plant related data were approximately normally distributed. Thus, the differences between treatments were determined using analysis of variance, and the least significant difference test (*P* < 0.05) used for multiple comparisons between treatments. One-way analysis of variance (ANOVA) was used to assess the significance of the variations of Cr among the different plant parts, followed by HSD tests. Graphical presentation was carried out using “Origin pro-2017”. Furthermore, the plots of principal component analysis on *B*. *napus* parameters were carried out by using the RStudio 4.3.1 software.

## 3. Results

### 3.1 Plant growth and biomass

In the present study, various growth parameters were also studied in *B*. *napus* grown in different levels of tannery wastewater (0, 33, 66 and 100%) under the application of Fe and Zn-lys. The results regarding various growth parameters are presented in Fig 1. According to the results, the maximum reduction in the growth (plant height, number of leaves, leaf area, root length) and biomass (fresh/dry weights of roots and leaves) of *B*. *napus* were observed at maximum level of tannery wastewater application (100%), compared to the plants grown in the control (without the addition of tannery wastewater). However, combined application of Zn and Fe-lys increased plant height, number of leaves, leaf area, root length, fresh weight of root, fresh weight of leaves, dry root weight and dry leaves weight by 33, 25, 40, 25, 32, 23, 40 and 29%, observed in the plants which were grown in 100% addition of wastewater in the soil, compared to those plants which were grown in 100% addition or irrigation wastewater without the application of Zn and Fe-lys.

The article "Combined application of zinc and iron-lysine and its effects on morpho-physiological traits, antioxidant capacity and chromium uptake in rapeseed (Brassica napus L.)" was retracted in 2022. Reasons: compromised peer review; a conflict of interest; concerns about the authorship.

**Fig 1:** Effect different levels of tannery wastewater on plant height (A), number of leaves (B), leaf area (C), root length (D), root fresh weight (E), root dry weight (F), leaf fresh weight (G) and leaf dry weight (H) under the application of Zn and Fe-lys on *B*. *napus*. Values are demonstrated as means of three replicates along with standard deviation (SD; n = 3). One-way ANOVA was performed and means differences were tested by HSD (*P* < 0.05). Different lowercase letters on the error bars indicate significant difference between the treatments. Different levels of tannery wastewater used are as follow: 0 (without irrigation with wastewater), 33 (33% irrigation with wastewater), 66 (66% irrigation with wastewater) and 100 (100% irrigation with wastewater).

### 3.2 Gas exchange parameters and chlorophyll contents

Gas exchange parameters, carotenoids and total chlorophyll contents of *B*. *napus* along with various levels of tannery wastewater treatments and with and without application of Zn-lys (10 mg/L) and Fe-lys (5 mg/L) are given in Fig 2. The addition of tannery wastewater significantly reduced the contents of chlorophyll, carotenoids, and gas exchange parameters of *B*. *napus*, in comparison to the plants under control treatment. A 100% application of tannery wastewater reduces the transpiration rate, stomatal conductance, net photosynthesis, water use efficiency, total chlorophyll, and contents of carotenoids by 68, 57, 62, 57, 76 and 60% respectively. Whereas, exogenous application of both Zn-lys (10 mg/L) and Fe-lys (5 mg/L) significantly (P < 0.05) improves gas exchange parameters, contents of carotenoids and total chlorophyll in *B*. *napus* even at all levels of tannery wastewater applications. As presented in Fig 2, all abovementioned characteristics of the plants were significantly improved by 46, 30, 30, 42, 34 and 31% respectively under the combined application of both Zn-lys (10 mg/L) and Fe-lys (5 mg/L) in plants irrigated with 100% tannery wastewater.

The article "Combined application of zinc and iron-lysine and its effects on morpho-physiological traits, antioxidant capacity and chromium uptake in rapeseed (Brassica napus L.)" was retracted in 2022. Reasons: compromised peer review; a conflict of interest; concerns about the authorship.

**Fig 2:** Effect different levels of tannery wastewater on chlorophyll contents (A), carotenoid contents (B), stomatal conductance (C), transpiration rate (D), net photosynthesis (E) and water use efficiency (F) under the application of Zn and Fe-lys on *B*. *napus*. Values are demonstrated as means of three replicates along with standard deviation (SD; n = 3). One-way ANOVA was performed and means differences were tested by HSD (*P* < 0.05). Different lowercase letters on the error bars indicate significant difference between the treatments. Different levels of tannery wastewater used are as follow: 0 (without irrigation with wastewater), 33 (33% irrigation with wastewater), 66 (66% irrigation with wastewater) and 100 (100% irrigation with wastewater).

### 3.3 Oxidative stress (electrolyte leakage, MDA and H_2_O_2_)

Various oxidative stress indicators i.e., MDA (malondialdehyde) contents, hydrogen peroxide (H_2_O_2_) initiation and electrolyte leakage (%) in the roots and leaves of *B*. *napus* plants were also measured (Fig 3). Results showed that increasing the concentration of tannery wastewater in the soil enhances the contents of MDA, H_2_O_2_ and EL (%) in the roots and leaves of *B*. *napus*, while the maximum increased in oxidative stress indicators was observed in the plants which were grown in 100% addition of tannery wastewater in the soil compared to the control treatment. Whereas, exogenous application of both Zn-lys (10 mg/L) and Fe-lys (5 mg/L) significantly (*P* < 0.05) mitigated the oxidative stress by lowering the contents of MDA, H_2_O_2_, EL in both leaves and roots of the plants as compared to the plants grown with zero application of Zn and Fe-lysine. At maximum concentration of tannery wastewater treatment combined with the application of Zn-lys (10 mg/L) and Fe-lys (5 mg/L) reduced the EL by 27 and 32% in roots and leaves of the *B*. *napus*, similarly contents of both MDA and H_2_O_2_ were declined by 20, 26, 32 and 39% in both roots and leaves of the plant as presented in Fig 3.

**Fig 3:** Effect different levels of tannery wastewater on MDA contents in the roots (A), MDA contents in the leaves (B), H_2_O_2_ contents in the roots (C), H_2_O_2_ contents in the leaves (D), EL percentage in the roots (E) and EL percentage in the leaves (F) under the application of Zn and Fe-lys on *B*. *napus*. Values are demonstrated as means of three replicates along with standard deviation (SD; n = 3). One-way ANOVA was performed and means differences were tested by HSD (*P* < 0.05). Different lowercase letters on the error bars indicate significant difference between the treatments. Different levels of tannery wastewater used are as follow: 0 (without irrigation with wastewater), 33 (33% irrigation with wastewater), 66 (66% irrigation with wastewater) and 100 (100% irrigation with wastewater).

The article "Combined application of zinc and iron-lysine and its effects on morpho-physiological traits, antioxidant capacity and chromium uptake in rapeseed (Brassica napus L.)" was retracted in 2022. Reasons: compromised peer review; a conflict of interest; concerns about the authorship.

### 3.4 Antioxidant enzymes activities

Activities of various antioxidants (superoxidase dismutase (SOD), peroxidase (POD), catalase (CAT) and ascorbate peroxidase (APX) were also measured from the roots and leaves of *B*. *napus* plants (Fig 4). The results illustrate that a significant decrease was observed in the activities of antioxidant enzymes i.e., SOD, POD, CAT and APX in the roots and leaves of the *B*. *napus* grown under different levels of tannery wastewater in the soil, compared to those plants which were not in the control treatment. Results also depicted the maximum decrease in the activities of antioxidant enzymes in the roots and leaves of the *B*. *napus* was observed in the plants grown in the 100% addition of tannery wastewater in the soil, compared to those plants which were grown in 0% addition of tannery wastewater in the soil. However, application of Zn and Fe-lys significantly (*P* < 0.05) increased the activities of SOD, POD, CAT and APX by 74, 57, 56 and 63% in leaves and 50, 47, 60 and 83% in roots of *B*. *napus*, compared to those plants which were grown without the application of Zn and Fe-lys (Fig 4).

**Fig 4:** Effect different levels of tannery wastewater on SOD activity in the roots (A), SOD activity in the leaves (B), POD activity in the roots (C), POD activity in the leaves (D), CAT activity in the roots (E), CAT activity in the leaves (F), APX activity in the roots (G) and APX activity in the leaves (H) under the application of Zn and Fe-lys on *B*. *napus*. Values are demonstrated as means of three replicates along with standard deviation (SD; n = 3). One-way ANOVA was performed and means differences were tested by HSD (*P* < 0.05). Different lowercase letters on the error bars indicate significant difference between the treatments. Different levels of tannery wastewater used are as follow: 0 (without irrigation with wastewater), 33 (33% irrigation with wastewater), 66 (66% irrigation with wastewater) and 100 (100% irrigation with wastewater).

### 3.5 Uptake and accumulation of Cr, Zn and Fe

The contents of Cr, Zn and Fe were also measured from the roots and shoots of *B*. *napus*, when grown in the different levels of tannery wastewater with or without the application of Zn and Fe-lys (Fig 5). Increasing the concentration of tannery wastewater in the soil induces a significant (*P* < 0.05) increase in the contents of Cr, while a significant decrease in the contents of Zn and Fe in the roots and shoots of *B*. *napus*, compared to control plants (Fig 5). Increasing levels of wastewater in the soil increased Cr contents by 53.3 in the roots and 22.5 times in the shoots of the plants grown in 100% addition of tannery wastewater in the soil, compared to the plants grown in the control treatment. Compared to the control treatment, the maximum decrease in the contents of Zn and Fe was 55 and 60% in the roots, while decrease by 50 and 75%, respectively in the shoots of *B*. *napus* plants under the irrigation of 100% wastewater in the soil, compared to the control treatment. Although, Cr contents were decreased by the application of Zn and Fe-lys and Cr contents decreased by 30% in the roots and 33% in the shoots in the plants grown in 100% addition of tannery wastewater in the soil, compared to the plants grown in the control treatment. In contrast, Zn and Fe contents were increased by the application of Zn and Fe-lys and were increased by 28 and 32% respectively in the roots and 31 respectively and 33% in the shoots in the plants grown in 100% addition of tannery wastewater in the soil, compared to the plants grown in the control treatment.

The article "Combined application of zinc and iron-lysine and its effects on morpho-physiological traits, antioxidant capacity and chromium uptake in rapeseed (Brassica napus L.)" was retracted in 2022. Reasons: compromised peer review; a conflict of interest; concerns about the authorship.

**Fig 5:** Effect different levels of tannery wastewater on the uptake/accumulation of Zn contents in the roots (A), Zn contents in the shoots (B) Fe contents in the roots (C), Fe contents in the shoots (D) Cr contents in the roots (E) and Cr contents in the shoots (F) under the application of Zn and Fe-lys on *B*. *napus*. Values are demonstrated as means of three replicates along with standard deviation (SD; n = 3). One-way ANOVA was performed and means differences were tested by HSD (*P* < 0.05). Different lowercase letters on the error bars indicate significant difference between the treatments. Different levels of tannery wastewater used are as follow: 0 (without irrigation with wastewater), 33 (33% irrigation with wastewater), 66 (66% irrigation with wastewater) and 100 (100% irrigation with wastewater).

### 3.6 Correlation analysis between growth, physiological traits and Cr uptake in *B*. *napus*

A Pearson’s correlation graph was constructed to quantify the relationship between various growth parameters with Cr uptake in different parts of the plant (Fig 6). Cr concentration in the roots was positively correlated with Cr concentration in the shoots, MDA contents, H_2_O_2_ initiation and EL, while negatively correlated with root length, plant height, transpiration rate, net photosynthesis, SOD activity in leaves, Zn contents in roots, carotenoid contents, stomatal conductance, APX activity in leaves, water use efficiency, POD activity in leaves, leaves fresh weight, root fresh weight, root dry weight, Fe contents in shoots, total chlorophyll contents, Fe contents in roots, POD activity in roots, number of leaves, leaf area, CAT activity in roots, SOD activity in roots, CAT activity in leaves, APX activity in roots and Zn contents in shoots. Similarly, Cr concentration in the shoots was positively correlated with Cr concentration in the roots, MDA contents, H_2_O_2_ initiation and EL while negatively correlated with root length, plant height, transpiration rate, net photosynthesis, SOD activity in leaves, Zn contents in roots, carotenoid contents, stomatal conductance, APX activity in leaves, water use efficiency, POD activity in leaves, leaves fresh weight, root fresh weight, root dry weight, Fe contents in shoots, total chlorophyll contents, Fe contents in roots, POD activity in roots, number of leaves, leaf area, CAT activity in roots, SOD activity in roots, CAT activity in leaves, APX activity in roots and Zn contents in shoots. This correlation is depicted a close connection between Cr uptake and growth in *B*. *napus*.

The article "Combined application of zinc and iron-lysine and its effects on morpho-physiological traits, antioxidant capacity and chromium uptake in rapeseed (Brassica napus L.)" was retracted in 2022. Reasons: compromised peer review; a conflict of interest; concerns about the authorship.

**Fig 6:** Correlation between morpho-physiological traits, Zn and Fe contents with Cr uptake in different parts of *B*. *napus*. Different abbreviations used in this figure are as follow: H_2_O_2_-R (H_2_O_2_ initiation in roots), H_2_O_2_-L (H_2_O_2_ initiation in leaves), CR-R (Cr contents in roots), MDA-L (MDA contents in leaves), CR-S (Cr contents in leaves), MDA-R (MDA contents in roots), EL-R (electrolyte leakage in roots), RL (root length), PH (plant height), TR (transpiration rate), NP (net photosynthesis), SOD-L (SOD activity in leaves), Zn-R (Zn contents in roots), Carot (carotenoid contents), SC (stomatal conductance), APX-L (APX activity in leaves), WUE (water use efficiency), POD-L (POD activity in leaves), LFW (leaves fresh weight), RFW (root fresh weight), RDW (root dry weight), Fe-S (Fe contents in shoots), Chl (total chlorophyll contents), Fe-R (Fe contents in roots), POD-R (POD activity in roots), NOL (number of leaves), LA (leaf area), CAT-R (CAT activity in roots), SOD-R (SOD activity in roots), CAT-L (CAT activity in leaves) APX-R (APX activity in roots) and Zn-S (Zn contents in shoots).

A heatmap-histogram analysis was also constructed to explore the relationship between the different growth attributes and Cr uptake (Fig 7). Only significant differences (aquamarine color) were observed in the Cr uptake for 100% addition of tannery wastewater in the soil and without the application of Zn and Fe-lys, while all other traits were showing non-significant differences (blue color) within the used treatments. This histogram depicted a clear difference between the Cr uptake abilities and growth attributes of *B*. *napus*.

The article "Combined application of zinc and iron-lysine and its effects on morpho-physiological traits, antioxidant capacity and chromium uptake in rapeseed (Brassica napus L.)" was retracted in 2022. Reasons: compromised peer review; a conflict of interest; concerns about the authorship.

**Fig 7:** Heatmap Histogram correlation between morpho-physiological traits, Zn and Fe contents with Cr uptake in different parts of *B*. *napus*. Different abbreviations used in this figure are as follow: LFW (leaves fresh weight), Fe-R (Fe contents in roots), MDA-R (MDA contents in roots), CR-R (Cr contents in roots), H_2_O_2_-R (H_2_O_2_ initiation in roots), H_2_O_2_-L (H_2_O_2_ initiation in leaves), MDA-L (MDA contents in leaves), EL-L (electrolyte leakage in leaves), EL-R (electrolyte leakage in roots), CR-S (Cr contents in leaves), RFW (root fresh weight), RDW (root dry weight), Fe-S (Fe contents in shoots), SOD-L (SOD activity in leaves), POD-L (POD activity in leaves), SOD-R (SOD activity in roots), Zn-R (Zn contents in roots), POD-R (POD activity in roots), Zn-S (Zn contents in shoots), LA (leaf area), Chl (total chlorophyll contents), PH (plant height), RL (root length), NP (net photosynthesis), CAT-R (CAT activity in roots), CAT-L (CAT activity in leaves), APX-R (APX activity in roots), TR (transpiration rate), SC (stomatal conductance), WUE (water use efficiency), NOL (number of leaves), Carot (carotenoid contents), APX-L (APX activity in leaves).

### 3.7 Principal component analysis

Principal component analysis (PCA) was used to evaluate the effect of different levels of tannery wastewater with the exogenous application of Zn and Fe-lys on different attributes of *B*. *napus* (Fig 8). Of all the main components, the first two components (Dim1 and Dim2) comprise more than 97% of the whole database and make up the largest portion of all components (Fig 8). Among this, Dim1 contributes 93.4%, and Dim2 contributes 3.6% of the whole dataset. In addition, Fig 8 also shows that Cr contents in roots and shoots, MDA contents, EL and H_2_O_2_ initiation in the roots and leaves were positively correlated in the dataset from all the variables. In contrast, Fe and Zn contents in roots and shoots, SOD, POD, CAT and APX activities in leaves and roots, morpho-physiological traits in leaves and roots, photosyntethic parameters and pigment contents were negatively correlated in the dataset from all the variables (Fig 8).

**Fig 8:** Loading plots of Principal Component Analysis (PCA) on different morpho-physiological traits, Zn and Fe contents with Cr uptake in different parts of *B*. *napus*. Different abbreviations used in this figure are as follow: LFW (leaves fresh weight), Fe-R (Fe contents in roots), MDA-R (MDA contents in roots), CR-R (Cr contents in roots), H_2_O_2_-R (H_2_O_2_ initiation in roots), H_2_O_2_-L (H_2_O_2_ initiation in leaves), MDA-L (MDA contents in leaves), EL-L (electrolyte leakage in leaves), EL-R (electrolyte leakage in roots), CR-S (Cr contents in leaves), RFW (root fresh weight), RDW (root dry weight), Fe-S (Fe contents in shoots), SOD-L (SOD activity in leaves), POD-L (POD activity in leaves), SOD-R (SOD activity in roots), Zn-R (Zn contents in roots), POD-R (POD activity in roots), Zn-S (Zn contents in shoots), LA (leaf area), Chl (total chlorophyll contents), PH (plant height), RL (root length), NP (net photosynthesis), CAT-R (CAT activity in roots), CAT-L (CAT activity in leaves), APX-R (APX activity in roots), TR (transpiration rate), SC (stomatal conductance), WUE (water use efficiency), NOL (number of leaves), Carot (carotenoid contents), APX-L (APX activity in leaves).

The article "Combined application of zinc and iron-lysine and its effects on morpho-physiological traits, antioxidant capacity and chromium uptake in rapeseed (Brassica napus L.)" was retracted in 2022. Reasons: compromised peer review; a conflict of interest; concerns about the authorship.

## 4. Discussion

Excessive discharge of Cr could be extremely toxic for normal plant growth, morphological and physio-biochemical processes and membrane integrity of plants [61]. Result of present study revealed that morphological traits of the plant including plant growth and biomass were significantly reduced through the addition of tannery wastewater in soil (Fig 1). Cr has the ability to decline the growth attributes as previously reported in different plants including *B*. *napus* [62], *Zea mays* [63], *Helianthus annuus* [64], and *Triticum aestivum* [65]. Cr toxicity can cause decrease in plant growth and biomass, as toxic concentration of Cr in the soil makes the uptake essential nutrients unavailable. This has been reported in various studies, i.e., *Brassica juncea* [66], and *Brassica campestris* [67]. In the present study, the application of Fe and Zn-lys considerable decrease Cr contents in different parts of the plants, which is also a main factor to decrease plant growth and biomass, when grown under different levels of tannery wastewater in the soil. Both Zn and Fe-lys are widely recognized as the amino-chelated fertilizers and they have the profound capacity to boost up the uptake of necessary nutrients and safeguard the plants against external stresses. Amino acids have shown tremendous potential of making complexes with different toxic metals and eventually reducing their mobility [11, 68]. In the present study, combined application of Fe and Zn-lys increased plant growth and biomass (Fig 1), which was also suggested by previous studies that an application of Zn or Fe-lys can be useful for increasing plant growth and biomass [22, 46, 47]. This is because Zn and Fe-lys enhances photosynthetic processes and provides a substantial growth in a short time under metal stressed environments [69].

The article "Combined application of zinc and iron-lysine and its effects on morpho-physiological traits, antioxidant capacity and chromium uptake in rapeseed (Brassica napus L.)" was retracted in 2022. Reasons: compromised peer review; a conflict of interest; concerns about the authorship.

Results revealed that gas exchange characteristics and chlorophyll contents of the *B*. *napus* were significantly reduced under the application of tannery wastewater. Cr toxicity in the soil caused a significant decrease in photosynthesis and contents of chlorophyll and carotenoids, which were also previously recorded in different plants such as *Zea mays*, *Oryza sativa*, *Spinacia oleracea* and *Helianthus annuus* [41, 63]. In the present study, a significant (*P* < 0.05) increased in the gas exchange characteristics and photosynthetic pigments of the *B*. *napus* were measured with the combined application of Zn and Fe-lys (Fig 2). Amino acids also take part in the increased leaf photosynthesis and thus increase of photosynthetic pigments of the plants [3, 70]. Results indicate that a combined application of both these micronutrients along with lysine effectively improves the gas exchange parameters and chlorophyll contents of the plants (Fig 2). Similar finding were reported by Rizwan et al. [11], and Bashir et al. [47] in *Triticum aestivum* and *Oryza sativa* (respectively) under Cd stress.

PTEs stress is a grave risk for plant growth, toxic concentration of HMs in plants and results in the over generation of reactive oxygen species (ROS) as compared to no stressed plants [15, 22, 71]. Increasing levels of tannery wastewater in the soil causes oxidative stress by over-production of ROS, which is manifested by increasing levels of MDA, H_2_O_2_ and EL in the roots and leaves (Fig 3). Previously, Cr toxicity induced oxidative damages in various organs of *Brassica juncea*, *Brassica oleracea botrytis*, and *Cymbopogon flexuosus* [41, 63, 72] have been reported. In our study, the application of Zn and Fe-lys significantly (*P* < 0.05) decreased the contents of MDA, H_2_O_2_ EL (%) in *B*. *napus* when grown in various concentrations of tannery wastewater and increased the activities of various antioxidant enzymes like APX, SOD, CAT and POD (Fig 4). It was noted that the application of amino acid chelation with micronutrients have ability to overcome the generation of ROS in the different parts of the plant. In addition, application of Zn or Fe-lys have ability to increase the activities of different enzymatic antioxidants, which was observed in soybean [73]. Similar results were also reported for *Oryza sativa* and *Spinacia oleracea* [22, 74]. However, the results are more promising that combined application of Zn and Fe-lys scavenges ROS generation (Fig 3), and offers a better option to enhance antioxidant capacity in various crops under wastewater treatments (Fig 4).

The article "Combined application of zinc and iron-lysine and its effects on morpho-physiological traits, antioxidant capacity and chromium uptake in rapeseed (Brassica napus L.)" was retracted in 2022. Reasons: compromised peer review; a conflict of interest; concerns about the authorship.

Our results stated that increases in the level of tannery wastewater application in soil resulted in significant accumulation of Cr contents in different parts of the plant by restricting the uptake of essential nutrients like Zn and Fe (Fig 5). High concentrations of Cr contents in different tissues of plants were also detected previously [22, 62, 75, 76]. The main effect of high concentrations of metals on the photosynthetic pigments and gaseous exchange parameters are related to decreases in the net photosynthesis rate, reduced ribulose-1,5-bisphosphate carboxylase/oxygenase (RuBisCo) efficiency, and the inhibition of electron transport and PSII activities [37, 77–79]. It was also observed that restriction in the uptake of necessary micronutrients is attributed to the inability of plants roots to successfully absorb these vital nutrients under the uncompromising stress of Cr toxicity [26]. This is because of the higher uptake of Cr in the plant parts significantly affects growth and composition of the plant [25, 30]. Although, our finding recommended that a combined exogenous application of Zn-lys and Fe-lys effectively restricts the accumulation and uptake of Cr and improved the accumulation of both Zn and Fe in various tissues of the plant (Fig 5). It was reported that, amino acids have ability to form complexes with different PTEs and results in immobilizing these metals and thus cause reduction in metal uptake by the plants [11]. In line with the result of this study, application of Zn-lys improves the concentration of Zn in various plants like *Triticum aestivum* [11], *Oryza sativa* [46] and *Spinacia oleracea* [22]. Similarly Fe-lys enhanced the contents of Fe in *Oryza sativa* [47] and *Zea mays* [63].

## 5. Conclusions

Our results confirmed that plant growth, photosynthesis and antioxidant system were adversely affected by Cr stress generated as a result of tannery wastewater application. Although, the oxidative stress and uptake/accumulation of Cr were enhanced with increasing levels of tannery wastewater applications. However, foliar application of Zn and Fe-lys improved plant growth and composition by decreasing the concentration of ROS and Cr concentration in various parts of the plants. Therefore, long-term field studies should be executed to draw parallels amongst plants/crops, metal stress, micronutrient fertigation regimes, nutrients mobility patterns and plant growth in order to gain insights into underlying mechanisms.

## Supporting information

S1 Table Physic-chemical properties of loam soil used in the pot experiment. (DOCX)

S2 Table Characteristics of tannery wastewater used for irrigation of the soil used in the pot experiment. (DOCX)
